RETRACTED

# Coupled Attention Framework of Convolutional Neural Network Based on Computer Intelligence

**DOI:** 10.1155/2022/7859287

**Published:** 2022-08-04

**Authors:** Huoxiang Yang, Yongsheng Liang, Wei Liu, Fanyang Meng, Chao Li

**Affiliations:** ^1^College of Electronic and Information Engineering, Shenzhen University, Shenzhen 518055, Guangdong, China; ^2^College of Computer, Shenzhen Institute of Information Technology, Shenzhen 518172, Guangdong, China; ^3^Hypermedia Communication Laboratory, Peng Cheng Laboratory, Shenzhen 518052, Guangdong, China

## Abstract

Using an attention mechanism based on the convolutional neural networks (CNNs) improves the performance of computer vision tasks by enhancing the representation of the features. The existing attention methods enhance the expression of the features by modeling the internal information of the features. However, due to the limited information flow of the previous features, these methods are difficult to calibrate features more completely. In this paper, we propose a Coupled Attention Framework (CAF) that is a simple attention framework for improving the performance of the existing attention methods. In the CAF, a coupling branch is added to an existing attention method to generate the input attention maps and enhance the input features of the convolution. The input attention is then spread to the output features through coupling between the input attention maps and convolution, the output features. The final result is the experimental results on various visual tasks. The results show that applying CAF to most of the existing attention methods can improve the performance with fewer parameters.

## 1. Introduction

The CNNs have been used in performing different visual tasks due to their powerful feature representation ability [1, 2]. To make features robust and increase the representation ability, several attention methods are designed to highlight the important semantic regions in the feature maps. This suppresses the possible semantic noise in the feature maps. The rapid development of the CNNs has motivated studies on the significance of the attention mechanism [3–6]. These empirical studies show that the attention mechanism can not only inform the important regions in the feature map but also enhance the expression of interest. The existing attention methods usually design a lightweight module that can be inserted into the basic CNN architecture. In recent research work, two important dimensions of feature maps, including space and channel, have been widely studied.

Based on the above two dimensions, the attention methods are divided into three categories: spatial and channel attention methods, spatial attention methods, and channel attention methods. Given any output features of a convolution layer, the attention extraction network of the attention methods infers the attention maps of the output features. Spatial and channel attention methods generate the 3d attention maps that can explicitly refine all positions of the features. However, the direct generation of the 3d attention maps is computationally complex, and the corresponding network is difficult to optimize. To overcome the above limitations, several methods utilize the attention mechanism to learn the channel attention and spatial attention separately from the channel dimension and spatial dimension. These methods have been rapidly developed due to their lower computational cost and the smaller number of parameters. When computing the attention maps from one dimension, the information of the other dimension is fully aggregated, and then using the aggregated features produces the attention maps. For example, the spatial information of the features is aggregated when inferring the channel attention maps. Generating a spatial context descriptor, the descriptor is then forwarded to an attention extraction network generating the 1D channel attention maps. The same applies to the channel attention maps where the 2D spatial attention maps are generated.

RETRACTED

For the past few years, investigations on the attention mechanisms in CNNs have been mostly focused on the performance improvement of one class of attention methods. To improve the performance of the attention methods and reduce the computational complexity, the design of exquisite attention models is challenging. To solve this problem, in this paper, instead of designing exquisite models for attention methods, we propose an attention framework that can improve the performance of the existing attention methods. We further propose a novel and efficient attention framework, namely, the Coupled Attention Framework (CAF) for the CNNs.

Taking a classical channel method SENet as an example, we describe how to apply the CAF to the SE method.  Figure 1(a) presents the overview of the existing SE method, and Figure 1(b) shows the application of the CAF to SE method. Here, *ξE* refers to the attention extraction network, which is the most important part of existing attention methods. The SE method first uses *ξE* extract attention maps by modeling the internal channel information of the output features. The channelwise features responses of output features are then adaptively calibrated by the channelwise multiplication between the attention maps and the features. To apply the CAF to the SE, CAF first generates input and output attention maps of the convolution layer by the attention extraction network. Then, the input attention is spread to the output feature maps by coupling of the input attention and the convolution. Finally, the output features are recalibrated by the output attention maps. Hence, the output feature maps receive multiscale attention information. Note that using the same attention network as in the SE method increases the computational costs and the number of parameters. To reduce the computational costs, we modify the last layer of the extraction network *ξE* to reduce the size of attention maps. Our experiments show that there is no performance loss compared with using the origin feature extraction network. Our method offers a fresh perspective on the performance improvement of the existing attention methods instead of designing exquisite models. The CAF is beneficial to both large-scale networks and lightweight networks. It is also suitable for applications such as object detection, image classification, and semantic segmentation tasks. Finally, this research contributes to a deeper understanding of attention mechanism in nonvisual studies.

RETRACTED

## 2. Related Work

Attention mechanisms aim to highlight the high-value semantic information and restrain the background noise. In this section, we will discuss the relevant research works on the three attention mechanisms mentioned.

### 2.1. Channel Attention Mechanisms

Here, the channel interdependence of the feature map is used to determine the attention map. One of the successful examples is SENet [7], which simply squeezes each 1D feature map to efficiently build interdependence among channels. SKNet [8] further introduces a dynamic kernel selection mechanism, which is guided by the multiscale group convolutions, with a small number of additional parameters and calculations to improve the classification performance. Later works, such as SRMNet [9], SPANet [10], and EPSANet [11], extend this idea by incorporating style information into the channel calibration or designing advanced pyramid-like structures. However, the realization of the channel interdependence heavily depends on the predesigned global average-pooling component, and hence these methods cannot emphasize informative regions in spatial because of missing spatial importance.

### 2.2. Spatial Attention Mechanisms

Here, the spatial importance of the feature map is used to calculate the attention map. BAM [12] and CBAM [13] use the spatial dimension for the purposes of reweighting in parallel or series, obtaining a superior performance while using the same parameters. From a lightweight point of view, SGENet [14] aims to improve the learning of different semantic subfeatures of each group. In every group, it generates a spatial attention map guided by the similarities between the global and local feature descriptors. Combining the advantages of the BAM and SGENet, SANet [15] improves the spatial distribution of each group by using shuffle operation and better performance against background noise. However, there are different informative parts in different spatial; one spatial attention map cannot express the importance distribution of all spatial on the feature maps.

RETRACTED

### 2.3. Channel and Spatial Attention Mechanisms

Here, the channel interdependence and spatial importance of the feature map are both used to calculate the attention map. The channel and spatial attention networks are recently very popular because they build the attention in spatial and channel. Typical examples include NL [16], A2Net [17], SCNet [18], GSoP-Net [19], and CCNet [20], all of which obtain attention information about the channel and spatial through nonlocal mechanisms. However, all these methods are heavy-weight, computationally inefficient, and hard to plug into multiple convolution layers.

Different from these approaches that leverage expensive and heavy nonlocal or self-attention blocks, our approach considers an attention framework that can improve the performance of the existing attention methods.

## 3. Methods

In this section, we first propose a unified mathematical formulation of the existing attention modules and analyze their limitation. The proposed attention framework, CAF, is then introduced in detail.

### 3.1. Problem Formulation

For any given input features *x* of a convolution layer, the convolution operator models the internal information of the input features and generates output features *x*′. Most of the existing attention methods calibrate *x*′ to generate the calibration features *y*. The above process can be formulated as follows:

(1) $$\begin{array}{c} x^{\prime }=F\left(x,w\right),\\ y=\xi E\left(x^{\prime }\right)⊙x^{\prime }. \end{array}$$

Here, ⊙ denotes elementwise multiplication. *F* refers to the convolution operation, and *w* ∈ *R*^*C*′×*C*×*K*_*h*_×*K*_*w*_^ denotes the convolutional filters with kernel size *K*_*h*_ × *K*_*w*_. *C*′ is the number of filters and *C* is the channel of filters. *ξE* refers to the attention extraction network, and *ξE*((*x*′)) denotes extracting the attention maps of *x*′. Here, *M* refers to the attention maps. Based on the corresponding attention extraction network, the generated attention maps can be broadly categorized into the following three types:

- *M* ∈ *R*^*C*×1×1^, where *ξE* belongs to the channel attention extraction network and generates the channel attention maps by utilizing the global context features aggregated by the context modeling module.
- *M* ∈ *R*^1×*H*×*W*^, where *ξE* belongs to the spatial attention extraction network and models the interspatial relationship of features to generate the spatial attention maps.
- *M* ∈ *R*^*C*×*H*×*W*^, where *ξE* belongs to the spatial and channel attention extraction network and generates the attention maps via modeling the spatial and channel information of the features.

RETRACTED

The existing attention methods generate the attention maps by modeling internal information of *x*′ to calibrate feature maps. However, lacking the information flow of the previous features *x* restricts the enhancement capability of the feature maps.

### 3.2. Coupled Attention Framework

To overcome the limitation mentioned above, we propose the CAF as follows:

(2) $$\begin{array}{c} x^{\prime }=F\left.\xi E_{1}\left.x\right\}⊗x,w\right\},\\ y=\xi E_{2}\left.x\right\}⊗x^{\prime }. \end{array}$$

Here, ⊗ denotes interpolation multiplication that we proposed. *ξE*_1_*x*} and *ξE*_2_*x*} denote two attention extraction networks applying on *x*. Comparing formulas (1) and (2), the main difference between them is that CAF has dual attention calibration on the output features. In CAF, *x* and *x*′ are both calibrated to enhance feature representation. Here, we first calibrate the input features *x*. Then, through the coupling of the input attention and convolution, the input attention information of the calibrated input is spread to the output features. The preliminary calibrated output features *x*′ are then generated. Finally, *x*′ are recalibrated to generate the final feature maps *y*. Note that we propose interpolation multiplication to reduce the costs of parameters and computation. In CAF, we modify the last layer of the existing attention extraction and present two key operations, including coupling and interpolation multiplication. In the following, each part of our module is presented in detail.

#### 3.2.1. Interpolation Multiplication

The existing methods calibrate the features by the elementwise multiplication between features and attention maps. In CAF, the last layer of attention extraction network is modified. The generated attention maps are lighter than the original maps, where channel attention *M* ∈ *R*^(*C*/*n*)×1×1^ and spatial attention *M* ∈ *R*^1×*H* × *W*}/*n*}^. Here, *n* > 1, and it is a hyperparameter used to reduce the number of parameters. As a result, we are unable to use elementwise multiplication to calibrate the features in CAF. To overcome the limitation of mismatch, we propose a simple interpolation multiplication. Interpolation method, also known as “interpolation method,” is to use the function *f*(*x*) to insert the function values of several points in a certain interval, make appropriate specific functions, take known values at these points, and use the value of this specific function as the approximate value of function *f*(*x*) at other points in the interval. This method is called the interpolation method. From the type of attention maps, the formula of interpolation multiplication can be expressed as follow: if *M* ∈ *R*^*C*/*n*}×1×1^,

(3) $$\begin{array}{c} {\tilde{x}}_{c}=\left\{\begin{array}{cc} x_{c}\times M_{a}, & c=a\times n,\\ x_{c}, & \text{others}, \end{array}\right) \end{array}$$

and if *M* ∈ *R*^1×*H* × *W*/*n*}^,

(4) $$\begin{array}{c} {\tilde{x}}_{s}=\left\{\begin{array}{cc} x_{s}\times M_{a}, & s=a\times n,\\ x_{s}, & \text{others}. \end{array}\right) \end{array}$$

*x*_*c*_ and *x*_*s*_ denote the feature sampled along the channel and spatial dimensions. $\tilde{x}$ refers to the calibrated features. As shown in Figure 2, the input attention information is first transferred to $\tilde{x}$ using the interpolation multiplication between input attention maps and input features. The input attention information is then spread to the output features by the following attention coupling.

RETRACTED

#### 3.2.2. Interpolation Multiplication

The red dotted box in Figure 3 shows the overview of attention coupling. For convenience, we simply use a convolution operation to implement the coupling function. In the realization of convolution, the input features are expanded into a *K*^2^ × *C*} × *H* × *W*} matrix, and the filters are expanded into a *C*′×*K*^2^ × *C*} matrix. The value of each position on the output features is accumulated by the value of *C* elementwise multiplication. As shown in the overview of the attention coupling, the red, blue, and green parts refer to the subfeatures with attention information. The input attention information of those subfeatures is firstly aggregated by the elementwise multiplication between subfeatures and filters. The aggregated information is then fused by the accumulation. After the above operations, the position of each point in the output features carries the input attention information. Therefore, the input attention information is spread to the output features by the attention coupling.

#### 3.2.3. Instantiations

We can integrate the proposed CAF into a standard architecture, such as ResNet blocks. The SE method is a classic attention method that can be used to improve the performance of ResNet. In order to introduce how to apply CAF to the attention method in detail, we introduce CAF-SE block in ResNet by applying CAF to the popular SE method. Note that bottleneck block is the building block for ResNet50/101, and basic block is for ResNet18/34. Figure 2 depicts the schema of CAF-SE block. For basic block, similar to SE, we apply CAF to the second 3 × 3 convolution. For bottleneck block, we also apply CAF to the 3 × 3 convolution instead of the last 1 × 1 convolution. Due to the limitation of paper length, the instantiations of applying CAF to other attention methods for networks are not presented here.

RETRACTED

## 4. Experiment and Analysis

In this section, we evaluate the performance of the proposed CAF from three different perspectives. Firstly, to test the generalization ability of CAF to visual tasks, three types of visual tasks were tested. Secondly, through the design experiments on large-scale (ResNet) and efficient (MobileNetV1 and MobileNetV2) networks, the effectiveness of different backbone networks is tested. Because ResNet involves two different building blocks, we chose two backbone networks: ResNet18 and ResNet50, including ResNet18 (including basic blocks) and ResNet50 (including bottleneck blocks). Finally, to investigate the generality of CAF for attention methods, it is applied to three attention methods with different types: SE (a channel attention method), SGE (a spatial attention method), and CBAM (a spatial and channel attention method). Note that *n* is set to 2 in this section.

### 4.1. Image Classification

We evaluate the performance of CAF on two benchmarks of image classification: Cifar100 [21] dataset and ImageNet [22] dataset.

#### 4.1.1. Cifar100

The Cifar100 dataset comprises a collection of 50k training and 10k testing pixel RGB images for 100 classes. During the training, images are randomly flipped horizontally and zero-padded on each side with four pixels before taking a random crop. The mean and standard deviation normalization are also applied. We train all the architectures from scratch by synchronous SGD with weight decay 5*e* − 4, momentum 0.9, and minibatch 128 for 200 epochs. The learning rate starts with 0.1 and decreases by a factor of 20 at the 60th, 120th, and 160th epochs. The networks with 18 layers are trained on 2 GPUs, whereas the networks with 50 layers use 4 GPUs.

For large-scale ResNet networks, we test CAF on ResNet18 and ResNet50 with different block. The results are shown in Table 1. For ResNet18, compared to the original attention methods, the methods with CAF outperform the comparative attention methods with considerable improvement, while the number of parameters and calculation cost are not increased. For the ResNet50, because of the special usage on bottleneck block, the methods with CAF have fewer parameters except for the SGE. For example, the SE method with CAF obtains a 0.63% accuracy increase with 2.37M reductions of parameters. For SGE with CAF, the accuracy is increased from 80.59% to 80.73% without any increase in the number of parameters and computation costs.

RETRACTED

For efficient networks, we validate the performance of CAF on the MobileNetV1 and MobileNetV2. The results are shown in Table 2. For SE and CBAM methods, applying CAF results in performance improvement and the reduction of parameters cost. For SGE with CAF, the accuracy of MobileNetV1 is increased by 0.35%, while the accuracy of MobileNetV2 is reduced by 0.01%. The reason for the poor effect of SGE with CAF might be attributed to the fact that CAF is not suitable for groupwise attention methods on the Cifar100 datasets.

#### 4.1.2. ImageNet

To verify the universality of the CAF on different datasets, we investigate the experiment results on the more challenging ImageNet dataset. The ImageNet 2012 dataset comprises 1.28 million training images and 50K validation images from 1k classes. We train the networks on the training set and report the accuracy on the validation set with a single 224 × 224 central crop. For data augmentation, we follow the standard practice and perform the random size cropping to 224 × 224 and random horizontal flipping. The practical mean channel subtraction is adopted to normalize the input images. All networks are trained with naive softmax cross without label-smoothing regularization. We train all the architectures from scratch by synchronous SGD with weight decay 0.0001 and momentum 0.9 for 100 epochs, starting from a learning rate of 0.1 and decreasing it by a factor of 10 every 30 epochs.

For ResNet18, the results are presented in Table 3. Similar to Cifar100, the attention methods with CAF are more efficient with the same number of parameters than the original forms. For the ResNet50 backbone, the attention methods with CAF perform well except for SGE. For SE and CBAM, the methods with CAF not only have fewer parameters but also have higher accuracy in the ImageNet classification.

For efficient networks, we report the results in Table 4. For MobileNetV1 and MobileNetV2, CAF provides lower performance when applied to the SE method. Nevertheless, the number of parameters of SE with CAF is fewer than that of SE. Compared with SGE and CBAM, these methods with CAF have fewer parameters and have higher accuracy in ImageNet classification.

From the above results, we can conclude that the CAF is not suitable for all the datasets and networks. However, it is effective in most cases of classification, especially for the improvement of basic block in ResNet.

### 4.2. Semantic Segmentation

For semantic segmentation tasks, we validate the CAF on the PASCAL VOC2012 dataset. Here, DeepLabv3 is selected as the base model due to its competitive performance. Due to the limitation of time and computing resources, we only examine CAF performance on the efficient networks MobileNetV1 and MobileNetV2. For a fair comparison, the experiments follow the settings of experiments on DeepLabv3. Our reimplementation follows every detail, including 16 batch size, 512 image crop size, 0.007 learning rate with polynomial decay, and 30K training iterations. The only difference is that we use multigrid (1, 1, 1) instead of (1, 2, 4). The results are shown in Table 5, applying that applying CAF to the existing attention methods substantially improves the results with almost the same computational cost.

RETRACTED

### 4.3. Object Detection

For the target detection task, we use SSDLite as the baseline method to verify CAF on PASCAL VOC2007 dataset. These models were pretrained on ImageNet and fine-tuned on PASCAL VOC2007. We followed the SSDLite official settings on their GitHub website. Starting from the learning rate of 0.001, the model was fine-tuned in 10 stages through synchronous SGD and reduced by 10 times in the seventh stage. The average accuracy (AP) values of the three methods were compared. As shown in Table 6, for all the attention methods checked, compared with the original network, the attention method using CAF improves the results. The above experiments show that the algorithm is suitable not only for classification tasks but also for semantic visual tasks.

## 5. Structures of CAF for Basic Block

The effectiveness of the proposed module is examined on the Cifar100 dataset. Unless otherwise specified, the attention mechanism is used in the second 3 × 3 convolution of residual block in ResNet18. Here, we mainly examine the SE method in this section.

### 5.1. Structures of CAF for Basic Block

In the basic block of CAF, we use a shared dimensionality-reduction layer to reduce the number of parameters. In this section, we take CAF-SE basic block as an example to assess the performance of different structures (as shown in Figure 4).  Table 7 summarizes the comparison results for different implementation. It is seen that ResNet blocks with the shared structure consistently outperform the no-shared structure. For example, the best result of no-shared structure achieves an accuracy of 78.29%, whereas the result of a shared structure achieves an accuracy of 79.00%. This 0.71% increase demonstrates that a network with a no-shared structure is more difficult to optimize.

The final design of the proposed CAF uses a shared structure as a dimensionality-reduction layer. Two convolutional layers are then applied in parallel to generate attention maps separately to fuse with input and output features.

RETRACTED

### 5.2. Attention to Different Features

To analyze the role of CAF and the way it affects the features, here we first examine the effectiveness of applying attention mechanism to input or output features. We then combine the two for comparison.  Table 8 shows that accuracy of 77.86% can be achieved by the ResNet18 alone, while applying the SE to the input features achieves an accuracy of 78.09%, an increase of 0.23%. When SE is applied to the output features, it achieves an accuracy of 78.11%, an increase of 0.25%, compared to the ResNet18. We find that it is slightly better than the result of SE (input), which means that attention to output features plays a more important role in the system performance. The effect of applying SE to both input and output features is also investigated on Cifar100. It is seen that it achieves an accuracy of 78.67%, exceeding ResNet18 by 0.81%, and outperforms other types of SE implementation. By applying CAF to SE, the CAF-SE method outperforms all other comparing methods.

We argue that the traditional methods of combining attention maps with output features miss the attention on input features. Therefore, the calibration effect of output features is limited. The results confirm that the method of applying the attention mechanism to input and output features is complementary to each other.

## 6. Conclusion

In this paper, we apply the attention mechanism to the existing attention methods and propose CAF. For a given input feature, the feature is input into the transform network to generate two attention graphs, which are fused with the input and output features at the same time. Then, the features are calibrated to improve the representation ability of CNN. Our experiments on two classification datasets, Cifar100 and ImageNet, verify the efficiency of CAF by comparing it with existing attention methods. On the basis of verification, it can effectively play an important role in future development, which is conducive to the development of research.

## Figures and Tables

**Figure 1:** (a) A channel attention method: SE method. (b) The overview of applying CAF to SE method.

**Figure 2:** SE and CAF-SE block in ResNet.

**Figure 3:** The overview of Coupled Attention Framework.

**Figure 4:** Structures of two designed CAF-SE blocks. (a) CAF-SE block with shared structure. (b) CAF-SE block with no-shared structure.

**Table 1:** Accuracy of ResNet methods on Cifar100.

Method	Acc (%)	Params (M)	FLOPs (G)
ResNet18	77.86	11.22	0.56
SE	78.11	11.31	0.56
CAF-SE	**79.00**	11.31	0.56
CBAM	77.94	11.31	0.56
CAF-CBAM	**78.25**	11.31	0.56
SGE	76.67	11.23	0.56
CAF-SGE	**77.17**	11.23	0.56

ResNet50	77.86	23.71	1.31
SE	80.18	26.26	1.32
CAF-SE	**80.81**	23.89	1.32
CBAM	80.12	26.26	1.33
CAF-CBAM	**80.63**	**24.06**	**1.32**
SGE	80.59	23.73	1.32
CAF-SGE	**80.73**	23.73	1.32

RETRACTED

**Table 2:** Accuracy of MobileNet methods on Cifar100.

Method	Acc (%)	Params (M)	FLOPs (G)
MobileNetV1	68.45	3.32	0.48
SE	68.69	3.80	0.49
CAF-SE	**69.63**	**3.68**	0.49
CBAM	68.65	3.80	0.49
CAF-CBAM	**68.94**	**3.68**	0.49
SGE	68.53	3.32	0.48
CAF-SGE	**68.88**	3.32	0.48

MobileNetV2	69.54	2.37	0.69
SE	69.73	2.94	0.70
CAF-SE	**70.44**	**2.46**	0.70
CBAM	69.75	2.94	0.70
CAF-CBAM	**69.81**	**2.46**	0.70
SGE	**69.85**	2.37	0.69
CAF-SGE	69.84	2.37	0.69

**Table 3:** Accuracy of ResNet methods on ImageNet.

Method	Acc (%)	Params (M)	FLOPs (G)
ResNet18	70.34	11.69	1.82
SE	71.14	11.78	1.83
CAF-SE	**71.52**	11.78	1.83
CBAM	71.34	11.78	1.83
CAF-CBAM	**71.56**	11.78	1.83
SGE	69.29	11.69	1.83
CAF-SGE	**70.30**	11.69	1.83

ResNet50	76.68	25.56	4.14
SE	77.18	28.09	4.15
CAF-SE	**77.56**	**25.89**	4.15
CBAM	77.63	28.09	4.15
CAF-CBAM	77.63	**25.89**	4.15
SGE	77.58	25.56	4.15
CAF-SGE	77.58	25.56	4.15

**Table 4:** Accuracy of MobileNet methods on ImageNet.

Method	Acc (%)	Params (M)	FLOPs (G)
MobileNetV1	72.56	4.23	0.59
SE	73.75	4.72	0.59
CAF-SE	**74.09**	**4.60**	0.59
CBAM	73.56	4.72	0.59
CAF-CBAM	**73.85**	**4.60**	0.59
SGE	73.67	4.23	0.59
CAF-SGE	**73.97**	4.23	0.59

MobileNetV2	71.82	3.50	0.33
SE	73.28	4.08	0.33
CAF-SE	**73.49**	**3.96**	0.33
CBAM	73.21	4.08	0.33
CAF-CBAM	**73.35**	**3.96**	0.33
SGE	73.15	3.50	0.33
CAF-SGE	**73.35**	3.50	0.33

**Table 5:** Semantic segmentation experiments on VOC2012.

Base model	Backbone	Mean IoU (%)
DeepLabV3	MobileNetV1 + SE	70.84
	MobileNetV1 + CAF-SE	**71.35**
	MobileNetV1 + CBAM	70.77
	MobileNetV1 + CAF-CBAM	**71.22**
	MobileNetV1 + SGE	70.69
	MobileNetV1 + CAF-SGE	**71.04**

DeepLabV3	MobileNetV2 + SE	71.36
	MobileNetV2 + CAF-SE	**71.94**
	MobileNetV2 + CBAM	71.42
	MobileNetV2 + CAF-CBAM	**72.21**
	MobileNetV2 + SGE	71.45
	MobileNetV2 + CAF-SGE	**71.80**

**Table 6:** Object detection experiments on VOC2007.

Base model	Backbone	AP (%)
SSDLite320	MobileNetV1 + SE	69.21
	MobileNetV1 + CAF-SE	**69.75**
	MobileNetV1 + CBAM	69.22
	MobileNetV1 + CAF-CBAM	**69.80**
	MobileNetV1 + SGE	69.18
	MobileNetV1 + CAF-SGE	**69.62**

SSDLite320	MobileNetV2 + SE	71.71
	MobileNetV2 + CAF-SE	**72.31**
	MobileNetV2 + CBAM	71.85
	MobileNetV2 + CAF-CBAM	**72.41**
	MobileNetV2 + SGE	71.69
	MobileNetV2 + CAF-SGE	**71.91**

**Table 7:** Effect of two structure of CAF on Cifar100.

Method	Share	Acc (%)	Params (M)
CAF-SE	×	78.29	11.34
CAF-SE	√	**79.00**	**11.31**
CAF-CBAM	×	78.01	11.34
CAF-CBAM	√	**78.25**	**11.31**
CAF-SGE	×	76.98	11.24
CAF-SGE	√	**77.17**	**11.23**

RETRACTED

**Table 8:** Effect of various SE and CAF-SE methods.

Method	Acc (%)	Params (M)
ResNet18	77.86	11.22
SE (input)	78.09	**11.26**
SE (output)	78.11	11.31
SE (input and output)	78.67	11.36
CAF-SE	**79.00**	11.31

## Data Availability

The data underlying the results presented in the study are available within the article.
